The article "Rat mRNA expression profiles associated with inhibition of ischemic acute kidney injury by losartan" was published in 2019. Journal: Biosci Rep.

# Rat mRNA expression profiles associated with inhibition of ischemic acute kidney injury by losartan

**DOI:** 10.1042/BSR20181774

**Published:** 2019-04-09

**Authors:** Yijin Wu, Wenying Peng, Ru Wei, Yanhe Zhou, Miaoxian Fang, Siyi Liu, Yujun Deng, Qi Yin, Xin Ouyang, Linhui Hu, Yating Hou, Chunbo Chen

**Affiliations:** 1 Department of Intensive Care Unit of Cardiac Surgery, Guangdong Cardiovascular Institute, Guangdong Provincial People’s Hospital, Guangdong Academy of Medical Sciences, 96 Dongchuan Road, Guangzhou 510080, Guangdong Province, P.R. China; 2 Department of Child Health Care, Guangzhou Women and Children’s Medical Center, No.9 Jinsui Road, Guangzhou 510623, Guangdong Province, P.R. China; 3 Forevergen Biosciences Center, Guangzhou 51000, Guangdong Province, P.R. China; 4 Department of Critical Care Medicine, Guangdong Provincial People’s Hospital, Guangdong Academy of Medical Sciences, 106 Zhongshan Er Road, Guangzhou 510080, Guangdong Province, P.R. China

**Keywords:** acute kidney injury, ischemia and reperfusion, losartan, mRNA, transcriptome

## Abstract

**Objective**: Losartan was reported to inhibit the progression of acute kidney injury (AKI), but little is known about the underlying pharmacological mechanisms. In the present study, the mRNA expression profiles in ischemic AKI rat kidney altered by losartan treatment were analyzed by next-generation deep sequencing technology.

**Methods**: Ischemia and reperfusion treatment was applied to induce AKI in Sprague–Dawley (SD) rats. The urea and creatinine contents in rat blood were measured. H&E staining was performed to evaluate the histological alteration of rat kidney tissues under a microscope. The TUNEL method was applied to analyze apoptosis in rat kidney tissues. The mRNA profiles in rat kidney were analyzed using next-generation deep sequencing. Differential gene expression was confirmed by quantitative qRT-PCR.

**Results**: The rat model of AKI induced by ischemia and reperfusion showed significant increases in urea and creatinine levels, accompanied by a disrupted kidney tubular structure and renal cell apoptosis. Losartan treatment effectively inhibited the changes in urea and creatinine, tubular structure, and apoptosis in AKI rat kidney. A large number of mRNAs were found to be differentially expressed in the kidneys of AKI rats treated with losartan, which are involved in multiple processes and signaling pathways. The expression of nine differentially expressed genes such as monocyte chemoattractant protein-1 (CCL2) and suppressor of cytokine signaling 3 (SOCS3) was confirmed by qRT-PCR and Western blot.

**Conclusion**: Losartan caused significant alterations in the gene expression profile in AKI rat kidney, which mediated its anti-AKI effects.

## Introduction

Acute kidney injury (AKI), also known as acute renal failure, is a common disease involving severe nephropathy featuring the characteristic of sudden dysfunction of the kidneys, which often develops in less than a week [1,2]. In a clinical context, AKI is common in hospitalized patients, and is associated with extremely high morbidity and mortality, especially in critically ill settings [3–6]. Previous etiological investigations showed that the severe impairment of kidney functions could be caused by multiple pathogenic conditions such as a significant decrease in blood supply in kidney tissues, toxicity due to exposure to hazardous reagents, various severe inflammation reactions, and also pathogenic occlusion of the urinary tract [7,8]. The progression of AKI is commonly accompanied by a number of severe complications including uremia, metabolic acidosis, body fluid imbalance, and chronic kidney disease (CKD) [1,9].

For the treatment of AKI, many therapeutic methods based on the specific causative factors have been applied in a clinical context, such as the use of liposomal amphotericin instead of amphotericin to treat fungal infections; moreover, obstruction relief was used to deal with obstructive AKI [3,10]. With the lack of efficient treatments, continuous renal replacement therapy or intermittent hemodialysis has been applied as the mainstay treatment to keep severe AKI patients alive [11]. Losartan is one of the effective inhibitors of angiotensin II (ANG II) type 1 receptors (AT1), which was approved for clinical usage in 1995. It has been widely used in the clinical management of various human disorders including diabetic kidney disease, high blood pressure, and multiple cardiac diseases such as acute myocardial infarction (AMI) [12–14]. Extensive investigations have revealed multiple mechanisms underlying the therapeutic effects of losartan, including the inhibition of sensitivity of the human organs to ANG II, promotion of the activity of plasma renin, the decrease in aldosterone release, and also the suppression of uric acid uptake [15].

At the molecular level, losartan could greatly alter the expression levels of key functional genes that are closely associated with disease progression. For instance, the expression of the integrity of gap junctions (GJs) and Peroxisome proliferator-activated receptor γ (PPARγ) coactivator 1α (PGC-1α) were found to be significantly repressed in ventricle tissues during the pathogenesis of AMI in male Sprague–Dawley (SD) rats [14]. However, the treatment with losartan greatly reversed the alterations in the expression of these two genes, which effectively inhibited cell death in the remote viable areas of rat ventricle after AMI onset [14]. Moreover, in the kidney tissues of spontaneously hypertensive rats, the application of losartan was shown to significantly change the expression levels of many functional genes including the nicotinamide adenine dinucleotide phosphate (NADPH) oxidase gene and the *Klotho* gene, finally resulting in marked inhibition of the typical renal pathological damage [16]. In addition, large-scale gene expression profile analysis also revealed that losartan could induce changes in the expression of a large number of genes while performing its therapeutic functions. In a next-generation sequencing-based transcriptome analysis, more than 1400 genes were identified as being significantly differentially expressed in a murine model of diabetes after treatment with losartan; these were shown to be involved in multiple biological processes (BPs) including endoplasmic reticulum stress and heat shock protein-related signaling [17]. These reports clearly showed that the alterations of key gene expression might be critical mechanisms mediating the various therapeutic effects of losartan, and gene expression profile analysis could be applied as a powerful method for the study of losartan pharmacology.

Notably, previous investigations also demonstrated that losartan has potential for treating AKI and CKD [18,19]. In one recent study using a murine AKI-CKD animal model, the AT1a receptor signaling pathway was established as one important factor in the development and mortality of AKI, and losartan effectively inhibited the increases in mortality, blood pressure, azotemia, and kidney fibrosis during the pathogenesis of AKI [19]. Losartan could also greatly suppress the development of CKD in rats with AKI, and significantly reduce the mortality following functional recovery after AKI [19]. However, the underlying mechanisms by which losartan acts on AKI progression, especially the alterations in gene expression that might be induced by losartan treatment, remain largely unknown. In the current study, we thus performed transcriptome-wide characterization of differentially expressed genes in a rat AKI model treated with losartan, to explore the molecular mechanisms associated with the inhibition of AKI progression by losartan.

## Materials and methods

### Animal grouping

The male SD rats used in the present study, in the age range of 6–8 weeks, and body weight range of 400–700 g, were obtained from the Guangdong Medical Laboratory Animal Center. The rats were kept in the Experimental Animal Center of Forervegen (Guangzhou, China) for 2 weeks before any experimental procedures were carried out. The SD rats for the experiments were raised in a standard breeding environment with a room temperature of 22°C and humidity of 55% under a 12:12-h light–dark cycle. Free access to standard food and drinking water was provided throughout the research period, and no fasting was performed before any experimental operations. In total, 18 SD rats were randomly categorized into the control group with no experimental treatments, the sham group, the groups with AKI induced by ischemia/reperfusion, and the losartan group treated with losartan after AKI induction. All the experimental procedures on SD rats were approved in advance by the Laboratory Animal Ethics Committee of Guangdong Provincial People’s Hospital.

### Establishment of the rat AKI model

The establishment of AKI in experimental SD rats was carried out in accordance with a previous report, with the following minor modifications [20]. Briefly, the rats were anesthetized with isoflurane and the rat retroperitoneal space was opened with a skin-deep incision. The vascular pedicles of both kidneys were mobilized, followed by rat bilateral renal artery occlusion with a microvascular clamp, which was maintained for 45 min. Subsequently, the rats were subjected to reperfusion treatment by removing the microvascular clamps; the reperfusion period was set to 24, 48, or 72 h. The SD rats used as the control group were raised under normal conditions and no surgery or additional treatments were performed on them. Another group of SD rats that underwent similar surgery and treatment, but no renal artery occlusion, was used as the sham group in the present study. The SD rats of the losartan treatment group were treated daily with 80 mg/kg losartan by intraperitoneal injection, for 7 days, before the surgical induction of AKI. Finally, the kidney tissues of SD rats were collected after the rats had been put under deep anesthesia, which were immediately used for the following analyses.

### Plasma urea and creatinine content determination

The urea and creatinine levels in rat blood plasma were measured as indicators of AKI development in the present study. Blood samples of approximately 2 ml were obtained from each experimental rat through the posterior orbital venous plexus after the reperfusion, as designated. The serum of each rat was collected by centrifugation at 4000***g*** for 15 min, which was then immediately used for the measurement of the levels of urea nitrogen and creatinine with a Roche Cobas C111 analyzer (Roche Diagnostics, International Ltd., Rotkreuz, Switzerland). For comparison of the urea nitrogen and creatinine amongst different groups of rats, the data from at least three biological replicates were used.

### Histopathological evaluation

After the SD rats had undergone AKI induction through ischemia and reperfusion, the kidneys of each rat were collected and washed with saline solution to remove blood. The rat kidneys were then fixed for 24 h in 10% formalin followed by embedding with paraffin; next, the kidneys were sliced into serial 2-µm-thick sections, which were then mounted on to the glass sides. The tissue injuries in rat kidneys were then evaluated using the kidney sections stained with Hematoxylin–Eosin. Under a microscope, the necrosis, swelling, and lysis of rat renal tubular epithelial cells were carefully analyzed to assess the rat kidney injury. Rat renal congestion and bleeding, as well as inflammatory cell infiltration, were also used as indicators of kidney injury.

### Cell apoptosis analysis

The TUNEL method was used to analyze the apoptosis of rat kidney cells in the present study using the One Step TUNEL Apoptosis Assay Kit (#C1088; Beyotime, Beijing, China), following the procedures recommended by the manufacturer. Briefly, the rat kidney tissue slides collected as described above were stained with TUNEL solution, 50 µl per slide, for 1 h at 37°C in the dark. Green fluorescence was used to specifically stain the apoptotic rat kidney cells, which were finally observed using a fluorescence microscope and photographed for comparison between different groups.

### Transcriptomic analysis and validation

Next-generation deep sequencing was used in the present study to compare the mRNA expression profiles between the rat kidney tissues from different groups, as previously described with minor modifications [17]. Briefly, total RNA samples from collected rat kidney tissues were extracted using TRIzol solution (Thermo Fisher Scientific, MA, U.S.A.), in accordance with the manufacturer’s instructions. Analysis with an Agilent 2100 Bioanalyzer (OD260/280) and agarose gel electrophoresis were performed to evaluate the quality of RNA samples. The cDNA library was generated from RNA samples of approximately 0.1 µg using the Clontech Smart PCR cDNA kit (#634925; Clontech Laboratories, Inc.), in accordance with the manufacturer’s instructions, followed by adaptor removal with RsaI digestion, and poly(A+) RNA amplification using low-cycle-number PCR and modified oligo(dT) primers. Subsequently, the cDNA samples were fragmented by sonication, profiled using an Agilent Bioanalyzer, and used for Illumina library preparation with NEBNext reagents (# E6040; New England Biolabs), followed by quality and quantity analyses with the Agilent Bioanalyzer 2100. The sequencing was performed using the Illumina HiSeq 2000 sequencing system, and the paired-end reads were generated and analyzed using the DNAnexus platform (DNAnexus, Inc.). The quantitation and differential expression of transcripts were completed using Cufflinks 2.0.2 software, in accordance with the RNA-Seq/3SEQ Transcriptome-Based Quantification.

Visualization in a genomic context was performed using the web-based DNAnexus viewer. The Gene Ontology (GO) analysis of differentially expressed genes was performed using the DAVID (Database for Annotation, Visualization, and Integrated Discovery) system, with a focus on the BPs, subcellular components, and molecular functions. The signaling pathways associated with these significantly differentially expressed genes were determined using the Kyoto Encyclopedia of Genes and Genomes (KEGG) method (http://www.genome.jp/kegg/). The differential expression of individual genes was confirmed by quantitative RT-qPCR using PrimeScript RT Master Mix (Takara, Dalian, China) and SYBR Real Time PCR Master Mix kit (Toyobo, Osaka, Japan), following the manufacturers’ instructions with the primers listed in Table 1.

**Table 1:** Sequences of primers used for quantitative RT-qPCR

Gene ID	Sequence (5′–3′)	Product length (bp)
R-Socs3-F	TCTTTACCACCGACGGAACC	124
R-Socs3-R	GTACCAGCGGGATCTTCTCG	
R-Wisp2-F	CAGTGGCTTGGAATGGAGGT	185
R-Wisp2-R	TCATGTCACCGTGTCCCTTG	
R-Pparg-F	TCTGGGAGATCCTCCTGTTGA	119
R-Pparg-R	CGAAGTTGGTGGGCCAGAAT	
R-Hmox1-F	TCTGCAGGGGAGAATCTTGC	135
R-Hmox1-R	TTGGTGAGGGAAATGTGCCA	
R-Myc-F	CTCTCCGTCCTATGTTGCGG	208
R-Myc-R	GAAGCCGCTCCACATACAGT	
R-Ccne1-F	CGGACACAGCTTCGGGTCT	120
R-Ccne1-R	ATCGGACTGAGAGGTCGGAG	
R-Ccl2-F	TGATCCCAATGAGTCGGCTG	217
R-Ccl2-R	GGTGCTGAAGTCCTTAGGGT	
R-Gpnmb-F	TGCCAACGGCAATATCGTCT	188
R-Gpnmb	TCCATTTCTTCCGTCCGTGG	
R-Fasn-F	GCATTTCCACAACCCCAACC	106
R-Fasn-R	AACGAGTTGATGCCCACGAT	
R-Col3a1-F	TGCAATGTGGGACCTGGTTT	214
R-Col3a1-R	GGGCAGTCTAGTGGCTCATC	
R-Gclc-F	GAGCGAGATGCCGTCTTACA	86
R-Gclc-R	TTGCTACACCCATCCACCAC	

### Western blot

Tissues resected from the rats subjected to the different treatments were ground on ice followed by lysis in RIPA buffer (Pierce, Rockford, U.S.A.). Proteins of the cell lysate were collected and quantitated using the BCA Protein Assay Kit (Pierce). Proteins were separated on 12% polyacrylamide gels and transferred to PDVF membranes (Millipore, MA, U.S.A.). After 1 h of incubation in 5% non-fat milk TBS, the membranes were exposed to suppressor of cytokine signaling 3 (SOCS3) (Cell Signalling Technology, MA, U.S.A., diluted 1:600) or MCP1/monocyte chemoattractant protein-1 (CCL2 )(Abcam, MA, U.S.A., diluted 1:5000) primary antibodies overnight at 4°C. Secondary antibodies Peroxidase AffiniPure Goat Anti-Rabbit IgG (H+L) (Jackson Immuno Research Labs, PA, U.S.A., diluted 1:4000; Abcam) were added to the membranes at room temperature for 45 min. Bands on the membranes were visualized using chemiluminescence reagent (Pierce). GAPDH (diluted 1:4000; Thermo Fisher Scientific) was used as an internal reference control. The relative expression of SOCS3 and CCL2 were quantitated using ImageJ software (http://imagej.nih.gov/ij/).

### Statistics

The SPSS 18.0 software package was used for the statistical analysis, and the significance of differences between groups was analyzed by analysis of variance (ANOVA). A *P*-value of <0.05 was used to define a significant difference.

## Results

### Ischemia/reperfusion induced rat AKI

To analyze the potential effects of losartan on the development of AKI, we first established the rat AKI model by ischemia and reperfusion, as introduced in the ‘Materials and methods’ section. In comparison with that in the sham group, the creatinine content in the plasma samples of rats after ischemia and reperfusion was significantly higher (Figure 1A). The highest degree of creatinine increase was observed in rats with reperfusion for 24 h (Figure 1A). The urea level in rat plasma was determined and also exhibited significant elevation after the establishment of AKI by ischemia and reperfusion (Figure 1B). Next, we performed histological analysis of rat kidney tissues, revealing clear swelling of renal tubular epithelial cells, with significant necrosis and cytolysis (Figure 1C). We also observed significant increases in renal interstitial congestion and bleeding in rat tissues after the induction of AKI, accompanied by inflammatory cell infiltration, compared with the findings in the sham groups (Figure 1C). Furthermore, using the TUNEL method, we found that ischemia and reperfusion induced a significant increase in apoptotic renal cells in rat kidney tissues associated with AKI, in comparison with the level in the sham group (Figure 1D). Taken together, these results indicate that severe AKI was induced by the I/R treatment in kidney tissues of experimental rats.

**Figure 1:** Rat AKI induced by ischemia and reperfusion (**A**) Plasma creatinine level in rats after AKI induction by ischemia and reperfusion treatment. The sham group was used as a control, and creatinine level was determined after reperfusion for 24, 48, and 72 h. (**B**) Plasma urea level in rats with AKI induced by ischemia and reperfusion treatment. (**C**) The structural changes in renal tubules of rats after ischemia and reperfusion treatment. H&E staining and microscopy were used to observe the histological properties. (**D**) Rat kidney cell apoptosis during AKI after ischemia and reperfusion treatment. Apoptosis was analyzed by the TUNEL method. *P<0.05. Abbreviation: I/R, ischemia and reperfusion.

### Losartan represses rat AKI

It was revealed in previous studies that losartan can potentially be applied as an inhibitor of the progression of AKI. To provide a further basis for its clinical application, the effects of losartan on AKI were here tested in our rat AKI model established by ischemia and reperfusion. We observed that the increase in urea content in rat plasma of the AKI group was greatly down-regulated by pre-treatment with losartan before model establishment, which was comparable with the level in the sham group (Figure 2A). Similarly, the plasma creatinine level in rats that underwent ischemia and reperfusion to induce kidney injury was also remarkably decreased by the treatment with losartan (Figure 2B). The inhibition of AKI progression by losartan was also evidenced by the obvious disappearance of abnormal histological features of rat kidney tissues after the application of losartan (Figure 2C). In addition, the apoptosis of renal cells in rat kidney tissues was markedly promoted by ischemia and reperfusion treatment, but was effectively inhibited by the pre-treatment with losartan (Figure 2D). The high significance of alterations in urea, creatinine, histological features, and apoptosis in AKI rats treated with losartan strongly suggested that losartan possesses great anti-AKI potential and might be applied as a novel drug for the clinical management of severe AKI. Further investigation of the underlying mechanism should provide a basis for future trials.

**Figure 2:** Ischemic rat AKI suppressed by losartan (**A**) Plasma urea content in AKI rats pre-treated with losartan. The sham group was used as a control. Urea levels were determined after reperfusion for 24, 48, and 72 h. (**B**) Plasma creatinine levels in rats treated with losartan followed with ischemia and reperfusion. (**C**) Regulation of rat renal tubular structure by losartan pre-treatment. H&E staining was carried out before the microscopy analysis. (**D**) Apoptosis of renal cells in AKI rat kidney suppressed by the administration of losartan. TUNEL method was performed to evaluate renal cell apoptosis. ^***^P<0.001 (compared with the sham group); ^+^*P*<0.05, ^++^*P*<0.01 (compared with the AKI group). Abbreviations: I/R, ischemia and reperfusion; LST, losartan.

### Losartan induces changes in the gene expression profile in AKI rats

To investigate the molecular mechanisms underlying the inhibition of AKI progression by losartan, we carried out a transcriptomic comparison using next-generation deep sequencing technology, to identify the genes significantly differentially expressed amongst the sham group, the AKI group, and the losartan group. In total, 422 genes were found to be differentially expressed between the sham group and the AKI group, including 226 up-regulated genes and 196 down-regulated ones. This showed the significant role of gene expression alteration in the pathogenesis of AKI (Figure 3A,B). In addition, a total of 195 genes were differentially expressed in the losartan group compared with their status in the AKI group, including 127 up-regulated genes and 68 down-regulated ones (Figure 3A,B). Notably, our hierarchical clustering analysis revealed that the majority of up-regulated genes in the AKI group were greatly down-regulated by the treatment with losartan, while the expression levels of most down-regulated genes in the AKI group were significantly raised by losartan (Figure 3A). The visualization of differentially expressed genes using volcano plots also demonstrated the significant alteration of gene expression profile between the sham and AKI groups, which was also greatly altered by losartan treatment (Figure 3B). In addition, we analyzed the distribution of significantly differentially expressed genes in the rat genome and observed that these genes were distributed on every chromosome except the Y chromosome (Figure 3C). We also observed similar genomic distributions of the differentially expressed genes between the AKI group and the losartan group (Figure 3C). The significant alteration of gene expression in the AKI group and losartan group indicated that abnormal changes of gene expression play roles in AKI development, which should be associated with the therapeutic effects of losartan on AKI progression.

**Figure 3:** Transcriptomic identification of differentially expressed genes induced by losartan (**A**) Hierarchical clustering of differentially expressed mRNAs induced by losartan in AKI rat kidney. The up- and down-regulated mRNAs in the heat map relative to the levels in the sham group are shown in red and green, respectively. (**B**) Volcano plot presentation of differential expression of mRNAs amongst the sham group, the AKI group, and the losartan group. (**C**) Genomic distribution of significantly differentially expressed genes induced by losartan treatment in AKI rat kidney after ischemia and reperfusion. Up-regulated genes are shown as red bars, and down-regulated ones as green bars. Abbreviation: LST, losartan.

### Functional categorization of differentially expressed mRNAs

For a comprehensive view of the BP and signaling pathways that might be regulated by losartan in AKI rats, these differentially expressed mRNAs were subjected to further bioinformatics analysis. We found by GO annotation that these differentially expressed genes regulated by losartan treatment in rat kidneys with AKI were distributed into multiple subcellular components including the envelope, extracellular regions, macromolecular complexes, membrane-enclosed lumen, and synapse (Figure 4A). In addition, differentially expressed genes were associated with a number of molecular functions, such as antioxidation, auxiliary transport, and as an electron carrier, enzyme regulator, molecular transducer, structural molecule, transcription regulator, and transporter (Figure 4A). Notably, we showed that losartan regulates the expression of genes linked to various BP, including anatomical structure formation, biological adhesion, cell killing and death, cellular component biosynthesis and organization, growth and developmental processes, immune system processes, metabolic processes, pigmentation, reproduction, responses to stimulus, rhythmic processes, and viral infection (Figure 4A). Furthermore, by KEGG annotation of the differentially expressed genes, we revealed that losartan could regulate the expression of key genes involved in distinct signaling pathways, such as transcription misregulation in cancer, tumor necrosis factor (TNF) signaling, pluripotency stem cell-regulating pathway, Ras signaling pathway, Rap1 signaling pathway, and PI3K-AKT signaling pathway (Figure 4B). The wide spectra of BP and signaling pathways associated with the genes induced to undergo differential expression by losartan suggested that losartan could regulate a complex molecular network to perform its anti-AKI roles.

**Figure 4:** Functional categorization of losartan-regulated differentially expressed mRNAs (**A**) Functional categorization of mRNAs differentially expressed in rat kidney after losartan treatment. Differentially expressed genes were categorized according to their GO BPs, molecular functions, and subcellular components. (**B**) Signaling pathways associated with differentially expressed mRNAs in rat kidney induced by losartan treatment. KEGG analysis was performed to evaluate the major signaling pathways regulated by losartan in AKI treatment.

### Confirmation of differential expression of genes

To support the reliability of our transcriptomic analysis, nine genes that were identified to be differentially expressed upon losartan treatment and are associated with inflammation and oxidative stress according to previous studies were further confirmed by RT-qPCR. We found that the expression levels of CCL2, Heme oxygenase 1 (HMOX1), SOCS3, and Glycoprotein non-metastatic b (GPNMB) were significantly elevated in rats after the induction of AKI by ischemia and reperfusion; however, their levels were remarkably suppressed by the treatment with losartan in rat kidney tissues (Figure 5A–C,E). In contrast, the expression of PPARγ and glutamate cysteine ligase catalytic subunit (GCLC) in rat kidneys was markedly down-regulated during AKI development, compared with the levels in the sham group (Figure 5F,G). The expression of these two genes was greatly elevated by losartan treatment in AKI rat kidney tissues (Figure 5F,G). In addition, the expression of WNT1-inducible signaling pathway protein 2 (WISP2), Type III procollagen (COL3A1), and Fatty acid synthase (FASN) were significantly suppressed in rats with AKI, but was not altered by the treatment with losartan (Figure 5D,H,I). Western blot confirmed that SCOS3 and CCL2 was up-regulated in the model rats but suppressed in the losartan-treated rats, which was consistent with the qPCR results (Figure 6). The changes in expression of the above genes were consistent with the results of transcriptomic analysis, which supported the reliability of our gene expressional profile data in the present study.

**Figure 5:** Validation of differentially expressed genes induced by losartan treatment Relative levels of nine genes, namely, *CCL2* (**A**), *HMOX1* (**B**), *SOCS3* (**C**), *WISP2* (**D**), *GPNMB* (**E**), *PPARg* (**F**), *GCLC* (**G**), *COL3A1* (**H**), and *FASN* (**I**), in the kidney tissues of rats with AKI and losartan treatment were confirmed by quantitative RT-PCR. β-Actin was applied as an internal standard for the relative quantitation of mRNA levels. *P<0.05; **P<0.01. Abbreviation: LOS, losartan. NS, no statistical significance.

**Figure 6:** Validation of the differentially expression of SOCS3 and CCL2 proteins induced by losartan treatment Western blot showing the expression of SOCS3 and CCL2 in the AKI model rats and the losartan-treated AKI rats. The expression of protein were quantitated by ImageJ software. ^++^*P*<0.01 (compared with the sham group); ^**^P<0.01 (compared with the AKI group).

## Discussion

AKI remains a severe renal disorder associated with high morbidity and mortality due to the poor understanding of its underlying pathogenic mechanisms and limited choices of therapeutic drugs for its clinical management [1,8]. Benefiting from the easy operation, low experimental cost, and short establishment period, rat AKI models constructed by ischemia and reperfusion surgery, also termed as ischemic AKI, have been widely used for both basic research on AKI’s pathogenesis and evaluation of the therapeutic roles of novel drug candidates [21–24]. As a widely used inhibitor of AT1, losartan has been considered a candidate drug for various human diseases including AKI and the ensuing CKD [18,19]. However, little is known about the pharmacological processes mediating the losartan-induced inhibition of AKI, especially the major BP and expression of key functional genes associated with cellular signaling networks. In the present study, we thus carried out a wide-spectrum characterization of differentially expressed genes using an AKI rat model established by ischemia and reperfusion, to explore the mechanism of AKI suppression by losartan; we placed special focus on the changes in the gene expression profile based on relative mRNA levels.

Consistent with previous reports [18,19], our analysis here showed that losartan significantly suppressed the development of acute injury of rat kidney tissues after ischemia and reperfusion treatment. Besides ischemia-induced AKI in kidney, losartan was also reported to inhibit the progression of other tissue injuries. For instance, ANG II generated in the local area of lung tissues was shown to promote acute lung injury induced by sepsis and acid aspiration, and the blockage of ANG II receptor by losartan greatly relieved the acute lung injury due to high-volume ventilation [25]. In addition, losartan could repress liver injury caused by ischemia/reperfusion via the regulation of PPARγg activation, which was widely established as a protective regulator of ischemia/reperfusion injury [26]. Moreover, losartan was also revealed as a repressor of myocardial ischemic/reperfusion injury [27], vascular injury induced by advanced glycosylation [28], brain injury [29], and endothelial damage associated with hypertension and type 2 diabetes mellitus [30]. Our finding of the inhibitory effects of losartan on the AKI rat model provided further evidence of the wide range of tissues regulated by losartan. The disclosure of the molecular mechanisms mediating these injury-regulating processes should provide novel insights into the pharmacological roles that losartan plays as a suppressor of tissue injury.

Gene expression profile analysis based on transcriptome-wide characterization using next-generation deep sequencing has recently been applied as a powerful method for research on the effects of therapies [31,32]. In the present study, we analyzed the mRNA profile in rat kidney with acute injuries caused by ischemia and reperfusion, as well as the changes in expression profile induced by losartan treatment in AKI rat kidney tissues. A large number of genes were identified to be differentially expressed in the AKI rat model and under treatment with losartan, which were involved in various BP and signaling pathways. For instance, our GO annotation revealed that multiple genes in rat kidney differentially expressed by losartan treatment were key genes regulating cell death and killing. It is well known that the acute tubular necrosis and ensuing abnormal loss of renal function is a major pathogenic mechanism of AKI [33]. The panel of cell death-related genes identified in our transcriptomic analysis might have played critical roles in acute tubular necrosis and other types of apoptosis closely related to AKI.

Our KEGG analysis also revealed many differentially expressed genes belonging to the major signaling pathways regulating cellular functions. The inhibition of Ras/ERK1/2 signaling was proven to be an effective method for protecting against AKI [34,35]. In the present study, we identified that many genes with differential expression induced by losartan treatment in rat kidney function in the Ras signaling pathway, suggesting that the regulation of Ras-related signaling activation might be a key molecular pharmacological mechanism of losartan in treating AKI. Moreover, the signaling cascades mediated by TNF-α (TNFα) act as a key mechanism of lung endothelial cell injury associated with AKI [36]. We also revealed that the expression of several genes involved in the TNFα signaling pathway was significantly altered in rat kidney tissues by losartan treatment, which indicated the critical roles that TNFα signaling might play during the losartan-induced suppression of AKI. In addition, the expression of nine genes in AKI rat kidney regulated by losartan treatment was further confirmed in the present study by quantitative RT-PCR, which was highly consistent with the transcriptome sequencing results. For example, CCL2, Hmox1, and SOCS3 are associated with inflammatory regulation. In SIRT2-deficient mice, the infiltration of neutrophils and macrophages, acute tubular damage, and decreased renal function after LPS induction were observed. During this process, the expression level of the inflammatory chemokine CCL2 in the mouse kidney was significantly down-regulated [37]. Damaged tubular epithelial cells release pro-inflammatory cytokines and chemokines, which help recruit immune cells. A bioinformatics analysis on the protein–protein interaction network regarding IR injury in the kidney in a previous study suggested that Hmox1 had the most nodes within this network. As IR injury is one of the causes of AKI, this indicates the involvement of Hmox1 in AKI [38]. Indeed, the cytoprotective effects of Hmox1 by modulating oxidative stress, autophagy, and inflammation have been well documented in AKI using an animal model and are considered to function as a therapeutic target of AKI [39]. SOCS proteins are important regulators of cytokine signaling that participate in maintaining balance in the immune system [40,41]. For instance, deletion of the suppressor of cytokine signaling 3 (*SOCS–3*) gene in mouse renal proximal tubules resulted in a great improvement and recovery of kidney function after AKI [42]. The identification of SOCS-3 in this study further highlighted the importance of this gene during AKI pathogenesis and treatment.

GCLC, GPNMB, and PPARγ have frequently been reported to regulate oxidant stress events. GCLC is a catalytic subunit of Glutamate cysteine ligase, and is closely associated with events following oxidative stress [43]. Studies have revealed that GCLC deficiency causes mitochondrial damage and neurodegeneration in a CNS mouse model [44] and leads to mitochondrial injury and hepatic failure [45]. Moreover, Vieira et al. [46] showed that the genetic variant GCLC rs17883901 is associated with an increased risk of renal disease in type 1 diabetes patients, suggesting its involvement in renal disease. PPARs are oxidative stress- and inflammation-associated ligand-activated transcription factors that have been shown to act as regulators of inflammation in ischemia-related and infectious diseases and insulin resistance [47–50]. The changes in expression of these inflammation- and oxidative stress-associated genes in the present study suggested the changes of inflammatory and oxidative stress-related processes upon treatment with losartan. Further study focussing on this perspective should provide more evidence on the precise pathological mechanism involved in AKI treatment with losartan.

In summary, in the present study we identified a large number of functional genes that were differentially expressed during the inhibition of AKI by losartan. Further functional investigations of these major genes in the context of AKI and losartan treatment should provide new perspectives on the pathogenesis of AKI, as well as on the pharmacological effects of anti-AKI candidates.

## Abbreviations

AKI: acute kidney injury
AMI: acute myocardial infarction
ANG II: angiotensin II
AT1: ANG II type 1 receptor
BP: biological process
CCL2: monocyte chemoattractant protein-1
CKD: chronic kidney disease
GCLC: glutamate cysteine ligase catalytic subunit
GO: Gene Ontology
GPNMB: glycoprotein non-metastatic b
Hmox1: heme oxygenase 1
KEGG: Kyoto Encyclopedia of Genes and Genomes
PPAR: peroxisome proliferator-activated receptor
SD: Sprague–Dawley
SOCS3: suppressor of cytokine signaling 3
TNF: tumor necrosis factor
